# Ameliorating Effects of Bioactive Peptides Extracted from *Litopenaeus vannamei* Wastes on Oxidative Stress, Glucose Regulation, and Autophagy Gene Expression in Nonalcoholic Fatty Liver-Induced Rats

**DOI:** 10.1155/2022/2679634

**Published:** 2022-08-25

**Authors:** Roya Moradian, Ebrahim H. Najdegerami, Mehdi Nikoo, Vahid Nejati

**Affiliations:** ^1^Department of Biology, Faculty of Science, Urmia University, Urmia, Iran; ^2^Department of Pathobiology and Quality Control, Artemia & Aquaculture Research Institute, Urmia University, Urmia, Iran

## Abstract

This study aimed to investigate the effect of bioactive peptides from *Litopenaeus vannamei* on oxidative stress, glucose regulation, and autophagy gene expression in the induced nonalcoholic fatty liver rats. Bioactive peptides used in the current study were extracted in a progressive rise in temperature (40–60°C) (GP). For this purpose, twenty-four healthy male rats (initial weight, 230.1 ± 22 g) were divided in four experimental groups including control (standard diet), HFD (high-fat diet), HFD + GP20, and 300 (high-fat diet + 20, 300 mg peptides/kg body weight). After 70 days, the results indicated that experimental treatments did not affect the body and liver weight (*P* > 0.05), although the higher liver weight was seen in HFD treatment. Based on these results, the use of GP peptides improved antioxidant enzymes and decreased MDA concentration, and a significant difference was observed between peptide treatments and HFD (*P* < 0.05). In comparison to the HFD group, significantly lower liver enzymes (ALT and AST) were seen in peptide treatments (*P* < 0.05). Also, the results indicated that the lowest amylase, alkaline phosphatase, glucose, insulin, HOMA-IR, and inflammation cytokines (TNF-ɑ and IL-6) were seen in peptide groups. The autophagy gene expression was measured in the liver cells, and the results showed that, unlike HFD treatment, the use of GP peptides decreased Beclin 1, Atg7, and P62 expression in male rat's livers. Overall, the results of the current study demonstrated that the use of GP peptides at low concentration shows significant hypoglycemia and antioxidant properties in nonalcoholic fatty liver-induced rats.

## 1. Introduction

Nonalcoholic fatty liver disease (NAFLD) is characterized in terms of the improper diet which is often associated with obesity, dyslipidemia, diabetes, hyperlipidemia, and hypertension and can progress to liver fibrosis, cirrhosis, and liver cell cancer [1, 2]. The factors such as gallbladder, intestine or stomach removal, pancreatic surgery, and using certain medicines can cause fatty liver disease. Thus, only a few therapies like lipid-lowering medications and insulin sensitizers were proposed to heal NAFLD. However, these medications have a series of adverse side effects, including weight gain, nausea, vomiting, and risk of mortality limiting their administration [3]. The side effects of chemical medicines have led researchers around the world to develop the techniques based on natural antioxidants and functional foods for health management and NAFLD control.

Oceans and marine environments are rich reservoirs of valuable products and provide important sources of bioactive compounds [4]. Among the industries related to the marine environment, aquaculture and fishing produce large amounts of protein-containing byproducts that can be hydrolyzed by commercial and microbial enzymes and produce bioactive peptides. Proteins hydrolysates or bioactive peptides contain 2 to 20 amino acids in their structure with a molecular weight of 200 to 1800 Da. The presence of particular amino acids and their location in the peptide chain dictates the bioactive properties of protein hydrolysates [5]. The physiological effects of protein hydrolysates such as immune stimulation [6], antimicrobial effects [7], antioxidant properties, cholesterol-lowering effects, [8] and antihypertensive effects [9] were reported in several studies. Based on these results, bioactive peptides were shown to regulate the complications of disorder in the patients with nonalcoholic fatty liver disease. Rite Vik et al. found that utilizing peptides isolated from salmon waste altered the fat metabolism of the liver, resulting in decreased fatty acid production and expression of lipogenic genes in the liver, as well as weight reduction in rats given these peptides [10]. A similar study by Huang et al. showed that the use of extracted oligopeptides reduces the secretion of liver enzymes ALT, AST, and MDA concentration in rats with nonalcoholic fatty liver [11]. Furthermore, Abbate et al. found that hydrolyzed wastes of anchovy fish reduced total cholesterol, serum triglyceride, liver enzyme activity, and hepatic acetyl glycerol [12].

Whiteleg shrimp (*Litopenaeus vannamei*) is known as the most important commercial species of shrimp at a rate of 5 million tons per year [13]. Since the waste production rate of 50% is related to this product, such a potential source for bioactive substances extraction can greatly assist the pharmaceutical industry [14]. Based on the aforementioned explanations and a huge amount of shrimp byproducts, this study aimed to investigate the effects of protein hydrolysates from whiteleg shrimp waste in a gradual process of increasing temperature (from 40 to 60°C) on oxidative status, glucose regulation, liver histopathology, and expression of genes related to autophagy in induced NAFLD male rats.

## 2. Materials and Methods

### 2.1. Peptide Preparation

To produce the protein hydrolysates, whiteleg shrimp wastes were minced with a meat grinder using a 3 mm hole plate (Pars Khazar Co., Tehran, Iran) and mixed with distilled water in a ratio of 1 : 1 and homogenized for 2 min (Heidolph Instruments GmbH, Schwabach, Germany). Nikoo et al. used a progressive rise in temperature (40–60°C, pH 7.1, over 3 h, 1°C rising every 9 min) to accomplish hydrolysis [15]. A mechanical stirrer was used to continually agitate the mixture throughout the enzymatic process. The solution was heated to 95°C for 10 minutes to cease the enzymatic process. After cooling and initial filtration by a mesh cloth, it was centrifuged at 4000 rpm for 15 min at 4°C. The supernatant was freeze-dried and stored at −20°C for further use. According to SEC-HPLC analysis, protein hydrolysates consisted of a high percentage of low-molecular-weight peptides (Figure 1). Dipeptides and tripeptides (180–500 Da) were the dominant peptidic fraction (64%) followed by free amino acids (MW < 180 Da; 27.4%). In general, 97% of peptides had MW less than 1 kDa. The percentage of peptides with MW > 3 kDa was only 1.7%.

### 2.2. Animals, Diets, and Experimental Design

Ten-weeks old, healthy male rats (initial weight: 230.1 ± 22 g) were obtained from the animal house of the Department of Biology (Urmia University, Iran). The rats (twenty-four rats) were fed within a standard diet during the adaptation period (25°C, 12–12 light/dark). After two weeks of adaptation to the experimental conditions, they were divided into four experimental groups (control; (HFD) high-fat diet (GP20), high-fat diet + 20 mg peptides/kg body weight (GP300), and high-fat diet + 300 mg peptides/kg body weight) and fed with the experimental diets for 70 days. Ten percent animal fat and 5% fructose were added to 85 percent of the regular meals to make the high-fat diet [16]. The bioactive peptide solution (20, 300 mg/kg body weight) was diluted in 4 ml distilled water and injected into the rats' stomachs through an oro-gastric feeding needle. 4 mL distilled water was delivered orally using an oro-gastric feeding needle in the control group. All animal experimental protocols were approved by the Animal Ethics Committee of Urmia University (N : IR-UU-AEC-3/1765/SC).

### 2.3. Blood Collection and Liver Sampling

At the end of the experiment, the rats were euthanized with an overdose anesthetizing of sodium pentobarbitone (90 mg/kg) to avoid undue stress during blood sampling and biopsy [17]. After weighing the animal, blood was drawn straight from the heart using 5 mm syringes loaded with a heparin anticoagulant. Plasma was isolated after centrifugation at 3500 rpm for 10 min and stored at −80°C to measure plasma biochemical indices and inflammatory cytokines (TNF-*α* and IL-6). After blood samples were taken, the rats' liver samples were weighed and separated into two portions for autopsy. A part was preserved at −80 degrees Celsius to assess oxidative stress, liver enzymes, and autophagy gene expression, while the remainder was fixed in 10% formalin for histological examination.

### 2.4. Biochemical Evaluations

#### 2.4.1. Measurement of Antioxidant Enzymes in the Liver

The liver kept at −80°C was used to measure antioxidant enzymes. For this purpose, 1 gr was mixed with physiological serum at a ratio of 1 : 10 and homogenized for 1 min (homogenization for 20 s with 5 s breaks). Then, the mixture was transferred to a microcentrifuge (20,000 rpm for 10 min, 4°C). The resulting supernatant was isolated and transferred to new microtubes for assessing total antioxidant activity (TAC), Reduced glutathione (GSH), Superoxide dismutase (SOD) enzymes, and malondialdehyde (MDA) concentration using commercial kits (Arsam Farazist kits, Urmia, Iran). Malondialdehyde (MDA) is measured to evaluate lipid peroxidation, which is one of the main cell damage indicators in animals and plants. TBARS test is a quantitative direct test to measure MDA. The samples and MDA control first react with TBA at 95°C. Then, a spectrophotometer of the samples and controls is performed after incubation. The rate of MDA is expressed in MDA nmol/mg of protein. TAC was measured using the ABTS technique. In the ABTS method, it is oxidized to ABTS + green in the presence of a suitable oxidant, which is blocked in the presence of an antioxidant. TAC can be measured by ABTS + absorption at 414 nm. The method described by Sun et al. [18] was used for SOD measurement where the activity of the enzyme is directly correlated with the degree of oxidation inhibition (Nitroblue tetrazolium) by the O_2_ anion. The absorbance was read at 580 nm, and the enzyme activity was expressed as a unit in mg of protein. The supernatant protein was determined by the Lowry [19] method using bovine serum albumin as a control.

#### 2.4.2. Measuring the Biochemical Indices and Proinflammatory Factors in Plasma

Commercial kits (Darman Faraz Kaveh, Isfahan, Iran) were used for amylase, alkaline phosphatase, liver enzymes (ALT, AST) as well as cholesterol and triglyceride measurements. The produced p-nitrophenol (read at 405 nm), which is directly correlated with the amylase activity, was used for amylase measurement and the activity was reported as U/ml. Alkaline phosphatase, which is colorless in a mildly acidic environment, isolates the phosphate group from 4-nitrophenyl phosphate to create 4-nitrophenol. In an alkaline environment, however, it generates a yellowish phenoxide ion that can be seen at 405 nm.

AST and ALT activity was evaluated in the plasma and the activity was reported according to kit's instructions (U/L). The triglyceride was measured based on the mechanism of its conversion to H_2_O_2_ by lipase, glycerol kinase enzymes, and glycerol phosphate oxidase. In the process, H_2_O_2_ produces a Quinoneimine colorful complex by peroxidase in the presence of 4-aminophenazone and 4-chlorophenol that can be read at 500 nm (mg/dl). The formation of the qunioneimine red-complex by H_2_O_2_ in the presence of 4-aminophenazone and 4-chlorophenol was used to measure total cholesterol content. The intensity of the color (OD = 520 nm) is proportional to the amount of serum cholesterol (mg/dl). At least, the levels of TNF-ɑ and IL-6 proinflammatory factors in the plasma were measured using Zelbio kits (Berlin, Germany) according to the manufacturer's instructions.

#### 2.4.3. Determinations of Fasting Blood Glucose, Glucose Tolerance, Insulin, and HOMA-IR

After 14 hours of fasting and access to water, the rats' fasting glucose levels and glucose resistance were determined [20]. A commercial kit was used to draw blood samples from the tail vein and assess the glucose content (Darman Faraz kave, Esfahan, Iran). To determine glucose resistance in the rats, glucose solution (2 g/kg body weight) was administered by gavage and blood glucose levels were measured at 0, 30, 60, 90, and 120 min using a glucometer, and the diagram of glucose changes was plotted for all trial groups at those time points. The following formula was used to calculate HOMA-IR : Insulin (*μ*IU/mL) × fasting glucose (*μ*mol/L)/22.5 [21]. The serum insulin level was measured using a kit by Zelbio Co. (Berlin, Germany) based on the ELISA technique.

### 2.5. Analysis of mRNA Expression of Autophagy Genes by RT-qPCR

TRIZOL method was used to evaluate the expression of the autophagy genes (Beclin 1, Atg7, LC3- ɪ, P62) in the rat's liver. For this purpose, 20–30 mg of liver tissue was homogenized using TRIZOL solution. The total RNA content was then extracted and measured using a nanodrop spectrophotometer to evaluate its quantity and purity (260 nm). For cDNA synthesis, RNA having a quality of greater than 1.8–2 was selected. The process was followed by cDNA synthesis according to the manufacturer's protocol (Pars Toos, CAT : A101161 Iran) in a 20 ml reaction mixture containing 1 mg RNA, oligo primer (1 *μ*L), a buffer (4 *μ*L), RNAse inhibitor (1 *μ*L), dNTP mixture 10 mM (2 *μ*L), and M-MuLV reverse transcriptase (1 *μ*l). Quantitative RT-PCR experiments for each sample were performed using a MyGo PCR (USA) thermal mini-cycler in three versions. qPCR reaction mixtures contained 0.5 *μ*l of cDNA pattern, 10 *μ*l of 2^×^SYBER GREEN master (High ROX, Noavarane Tebe Beynolmalal, Iran), and 0.5 *μ*l of forward and reverse primers of target genes (Table 1). Special primers were designed and produced by Gene Fanavaran Co. (Tehran, Iran) using a “multiple alignment program for amino acid or nucleotide sequences” (MAFFT, V.7) (https://maﬀt.cbrc.jp/alignment/server). The primer pair sequences for each gene are presented in Table 1. The qPCR thermal cycling conditions were as follows: a general denaturation process at 95°C for 5 min followed by 40 denaturation cycles at 95°C for 20 s, annealing at 72°C for 30 s. Mean values of cycle threshold (CT) from triple readings of each gene were normalized considering the mean CT values of the internal control gene (GAPDH) and the relative expression levels of the aforementioned genes were calculated using the ΔCt method: 2^−(dCt gene of interest − dCt internal control gene)^ [22].

### 2.6. Liver Tissue Preparation and Analysis

Histological studies of the liver were performed on samples fixed in a 10% formalin solution. Fixation, drying, tissue passage, paraffin blocks, and 5-microns slices were all completed after the fixation, drying, and tissue passage processes. The amount and quantity of fat vacuoles were next evaluated under a light microscope after staining sections with hematoxylin and eosin and Sudan Black [23].

### 2.7. Statistical Analysis

All data are expressed as mean ± standard division (SD) for *n* = 3 rats per treatment. The values were examined for normality (Kolmogorov–Smirnov test) and homogeneity of variance (Levene's test), then one-way ANOVA and Kruskal–Wallis tests were used to compare the means. Excel 2013 was used to draw the graphs and SPSS software V.21 was applied to examine statistical changes in experimental treatments.

## 3. Results

### 3.1. Weight Gain and Relative Weight of the Liver

The results of the effects of GP peptides on the weight gain and relative weight of the liver are presented in Table 2. The findings revealed that the rats fed on experimental diets had no significant difference in case of weight gain and relative weight of the liver (*P* > 0.05). Although the lowest and highest values for weight gain and relative weight of liver were observed in HFD treatments, respectively.

### 3.2. Oxidative Status in the Liver and Serological Parameters

Figure 2 depicts oxidative status (TAC, SOD, GSH, and MDA) in the liver of the control and the others. As expected, the rats fed on HFD showed a significant decrease in TAC, GSH, and SOD activity and a marked increase in MDA concentration which differed from other treatments (*P* < 0.05). Also, the results indicated that the GP peptides' administration (HFD + FP20, HFD + FP300) significantly increased TAC in the rats when compared with HFD (*P* < 0.05). The rats fed on HFD + FP20 showed a significant increase in SOD activity in comparison with HFD (*P* < 0.05). No significant difference was observed between HFD + FP300 and HFD (*P* > 0.05). Furthermore, as presented in Figure 1, GP administration in both doses significantly decreased MDA concentration when compared to HFD (*P* < 0.05). The rats fed on HFD + FP20 showed a significant increase in GSH which differed from other treatments (*P* < 0.05). No significant difference was seen between HFD + FP300 and HFD (*P* > 0.05).

Data in Figure 3 exhibit the effect of the GP peptides extracted from whiteleg shrimp waste on serum triglyceride and cholesterol. The results indicated that the rats fed on HFD and GP peptides had a significantly higher cholesterol content than the control (*P* < 0.05). Also, the results showed that the lowest triglyceride concentration was seen in GP peptides treatments between differed HFD and control groups (*P* < 0.05). Based on these results, it can be observed that triglyceride was significantly elevated in the HFD group as compared to the control (*P* < 0.05).

The plasma alkaline phosphatase and amylase activities were evaluated in the experimental treatments and the results are presented in Figure 4. As expected, HFD-fed rats showed a significant increase in serum amylase activity when compared to other treatments (*P* < 0.05). No significant difference was seen between control and GP peptides treatments (*P* > 0.05). Also, the findings revealed that the rats fed on control and HFD + GP20 had a significantly lower alkaline phosphatase activity as compared to HFD and HFD + GP300 treatments (*P* < 0.05). Furthermore, the highest value for alkaline phosphatase was observed in HFD which significantly differed with HFD + GP300 treatment (*P* < 0.05).

### 3.3. ALT, AST, and Proinflammatory Cytokines

Figure 5 exhibits the data of serum ALT, AST, and AST/ALT ratio as affected by GP peptides. The level of ALT and AST increased significantly when the rats fed on HFD as compared with GP peptides treatments (*P* < 0.05). The lowest values for the aforementioned parameters were observed in control which differed with GP peptides groups (*P* < 0.05). The AST/ALT ratio is an important index in the diseases related to fatty liver and based on our results, the rats fed on HFD exhibited a significantly higher ratio as compared to those fed on others (*P* < 0.05).

The results of the effects of GP peptides on plasma proinflammatory cytokines are presented in Figure 6. Our results showed that the GP peptides showed an anti-inflammatory potential and the lowest value for TNF-ɑ was seen in HFD + GP20, HFD + GP300 and control, respectively (*P* < 0.05). As expected, the highest level of TNF-ɑ was observed from HFD which had a significant difference with other groups (*P* < 0.05). In addition, IL-6 levels changed in experimental groups, and in contrast to HFD, the rats fed on GP peptides had a significantly lower IL-6 level (*P* < 0.05).

### 3.4. Effects on Fasting Glucose, Glucose Tolerance, Insulin Secretion, and HOMA-IR

Plasma concentrations of fasting glucose, insulin, glucose tolerance, and HOMA-IR are presented in Figure 7. The results indicated that the rats fed on HFD had the highest plasma fasting glucose value in comparison with the other treatments (*P* < 0.05). No significant difference was seen between the control and GP peptide groups (*P* > 0.05). Insulin concentration was higher in HFD and no significant difference was found between HFD and GP peptides (*P* > 0.05), although the lower values were seen in the rats fed on GP peptides. The plasma concentration of insulin in control and GP peptides did not show a significant difference (*P* > 0.05). Also, the results indicated that HFD increased glucose tolerance while GP peptides extracted from whiteleg shrimp decreased the aforementioned parameter in the rats. The lowest glucose tolerance was observed in the control treatment.

### 3.5. Effects on HFD and GP Peptides on the Expression of Liver Autophagy Genes

To find the effects of dietary treatments on autophagy gene expression, the alterations of Becline 1, Atg7, LC3-ɪ, and P62 expression were investigated in the liver (Figure 8). At the end of the experiment, the results indicated that the highest expression of Becline 1 was seen in HFD, control, and finally in GP peptides treatment which was significantly different (*P* < 0.05). Dietary treatments affected Atg7 expression and the rats fed on GP peptides showed the lowest expression in comparison with HFD and control (*P* < 0.05). The expression in HFD + GP20 was significantly lower than in the high dose (*P* < 0.05). Feeding on HFD + GP20 significantly increased LC3-ɪ expression when compared to the others (*P* < 0.05). No significant difference was found between HFD and high doses of peptides (*P* > 0.05). A significant increase of P62 expression was seen in HFD which differed from the others (*P* < 0.05). There was no significant difference between GP peptides and control (*P* > 0.05).

### 3.6. Histological Examination

The hematoxylin and eosin and Sudan black staining results of liver tissue are shown in Figures 9 and 10. Based on both staining results, the rats fed on the control diet exhibited normal morphology while HFD-treated rats had more lipid vacuoles than other treatments and the appearance was looking like the fatty liver. Also, the results indicated that oral administration of GP peptides exhibited a beneficial effect on the histological examination of livers. The livers of all GP peptide treatments were ameliorated and emerged with less lipid infiltration of hepatocytes as compared with HFD treatment.

## 4. Discussion

Nowadays, natural antioxidants such as bioactive peptides are used to improve NAFLD. GP peptides from whiteleg shrimp wastes which were extracted in a process by increasing temperature (40 to 60°C) were used to improve NAFLD complications in the rats. The results showed that GP peptides improved oxidative status, inflammatory factors, liver histopathology, and regulated the expression of autophagy genes in hepatocytes.

Body and liver weight did not affect by experimental diets, although respectively the highest and lowest values for the aforementioned parameters were seen in HFD group. HFD's palatability and high energy content seem to have lowered food intake and, as a result, weight loss in rats [16]. The findings on body and liver weight are consistent with the rats' liver histology and oxidative state.

Using GP peptide improved fasting glucose, insulin, and glucose tolerance in NAFLD-induced rats. Numerous studies have shown the inhibitory effects of bioactive peptides on glucose and insulin release. Based on these findings, bioactive peptides decrease the activity of digestive enzymes and fat buildup in the liver, lowering glucose absorption, insulin secretion, and the synthesis of proinflammatory markers in the liver [20, 24]. The inhibition effect on proinflammatory factors decreases insulin resistance and stimulates insulin signaling [20]. Moreover, Das et al. indicated that taurine has a hypoglycemic effect and decreases glucose uptake and insulin secretion [25]. To the best of our knowledge, taurine is an amino acid that is abundant in fish meal, but limited in plant protein sources [26]. In contrast, Drotningsvik et al. showed that the obese rats fed on cod, herring, and salmon protein had a lower glucose tolerance whereas fasting glucose and insulin concentration did not change [27, 28]. When compared to the HFD therapy, the findings showed that GP peptides dramatically reduced fasting hyperglycemia, insulin secretion, and proinflammatory markers. The peptide treatments caused higher glucose depletion than the insulin treatments, showing that glucose was decreased in mechanisms other than insulin production. HOMA-IR index is widely used to evaluate insulin resistance in animal models and humans [29, 30]. The rats fed on GP peptide showed lower HOMA-IR, indicating insulin resistance improvement which is the main pathological phase in the progress of dyslipidemia and NAFLD [31, 32].

Bioactive peptides are capable of inhibiting lipid accumulation in induced NAFLD animals [28, 33, 34]. The results indicated that the rats fed on HFD had higher triglycerides while feeding on GP peptides lowered triglycerides. These findings were supported with other studies that indicated bioactive peptides by regulation enzymes involved in triglyceride synthesis, lipoprotein lipase activity, fatty acid oxidation, and liver enzymes decrease triglyceride in plasma [35, 36]. Supplementation with GP peptides reduced cholesterol levels in rats, according to the findings. High cholesterol levels may lead to liver cell malfunction, NAFLD, and cardiovascular disease [37]. The obtained results are consistent with histological observation and indicate that GP peptides improve lipid accumulation in the rats fed on HFD (HFD + GP20, 300).

Oxidative stress occurs in the tissues which cause the development of metabolic syndrome in NAFLD rats [38]. Reactive oxygen species (ROS) are produced by a variety of processes, resulting in oxidative stress. One source of ROS is lipid buildup and oxidation, which causes liver cell inflammation and apoptosis. Another mechanism of producing ROS is the high consumption of oxygen by the mitochondrial respiratory chain, which occurs in terms of oxidative phosphorylation [39, 40]. Mitochondrial disorders caused by lipid peroxidation leads to MDA synthesis as one of the oxidative and tissue damage markers in the liver [41]. In the current study, MDA concentration increased in the rats fed on HFD which is consistent with previous reports that high-fat diets elevate oxidative indicators [42, 43]. Due to a rise in free radicals in hepatocytes, the levels of other antioxidant indicators including SOD, TAC, and GSH reduced as the quantity of MDA rose. Our results indicated that using GP peptides reduced MDA concentration and increased SOD activity, TAC, as well as GSH levels. Several studies reported that bioactive peptides reduce stress levels in different cells using various mechanisms including free radical scavenging, chelating, production of stable products with an electron donor, and finally increasing the expression of some genes involved in oxidative stress [44, 45]. Ultimately, these functions reduce oxidative stress and MDA concentration.

Oxidative stress and lipid peroxidation-mediated cell damage and stimulate the liver indicators enzyme activities. As a result of liver cell damage, the concentration of liver enzymes (ALT, AST), amylase, and ALP increase in plasma [42]. ALP is a membrane hydrolysis enzyme that is used as a biomarker for cholestasis, which is caused by hepatic steatosis and a lipid-carbohydrate metabolic imbalance [46, 47]. An increase above parameters stimulates proinflammatory cytokines (TNF-ɑ and IL-6) in the bloodstream, resulting in reduced lipid degradation and increase accumulation [48]. Feeding on GP peptides caused a significant decrease in the ALT, AST, amylase, ALP, and proinflammatory cytokines when compared with HFD treatment. Lower lipid accumulation in hepatocytes of the 6 rats receiving GP peptides was indicated in this study (histological images, Figure 9). It was indicated the inhibitory effects of these peptides on hepatic fat accumulation and consequent reduction in inflammatory factors and thus alkaline phosphatase.

In alcoholic and nonalcoholic fatty liver disease, autophagy is one of the cell's defensive mechanisms against pathological circumstances [50]. It may be inferred that raising the expression of these genes in response to intracellular stress decreases the rate of apoptosis, allowing injured cells to survive and be preserved [22]. To make a clear conclusion about stress oxidative and lipid accumulation in the hepatocytes, expression levels of autophagy-markers (Beclin-1, Atg7, LC3-ɪ, P62) were evaluated in the liver. In autophagy, initially, Beclin-1, the main regulator, forms a double membrane structure called the autophagosome. In the next step, Atg7 in collaboration with other proteins joins in the lipid conjugation of LC3-ɪ and membrane elongation [51]. Ultimately, the LC3-II is produced from LC3-I to complete the autophagosome formation [52]. To complete this puzzle, P62 as a reporter, transfers damaged cargoes for autophagy [53]. Also, P62 by self-transcription or/and in interaction with nuclear factor-erythroid factor 2-related factor 2 (Nrf2) retains autophagy starting in oxidative status [54]. In the current study, the rats fed on HFD showed the highest lipid peroxidation and proinflammatory factors indicating oxidative stress in the cells. Also, the highest Beclin 1 and P62 expression level was observed in this group indicating a huge deposition of damaged cargo. It seems HFD induces oxidative stress, and thus, the autophagy process initiates through Beclin 1 and P62-independent or/and dependent signaling [54, 55]. In line with previous results, the rats fed on GP peptides did not show a higher expression level of the aforementioned genes, most probably indicating the lower deposition of aggregated cargos. Also, the expression level of Atg7 in experimental treatments was lower than in the control, indicating the Atg7 expression is not synchronous with Beclin 1 and P62, which can eventually stop autophagy and apoptosis in the hepatocytes.

## 5. Conclusion

The HFD caused hyperglycemia and an increase in oxidative stress, according to the present research. Eliminative autophagy is most likely shown by changes in metabolomics and biochemical markers. In NAFLD-induced rats, the GP peptides isolated from *Litopenaeus vannamei* wastes, on the other hand, improved oxidative state, inflammation, liver enzyme activity, and glucose intolerance. Following the reduction of oxidative stress and other biochemical markers associated with NAFLD, the expression of autophagy genes decreased in GP peptide treatments. Based on these results and nutritional proprieties, GP peptides at low concentration could be used as a useful nutritional strategy in NAFLD treatment and prevention.

## Figures and Tables

**Figure 1:** Molecular weight distribution (MWD) of protein hydrolysate from *Litopenaeus vannamei* wastes by Alcalase enzyme. Substrate ratio was 5% for 180 min in a process with increasing temperature (40 to 60°C).

**Figure 2:** Effects of oral administration of GP peptides on the content of TAC, MDA, GSH, and SOD activity in liver tissues of the rats fed on experimental treatments. Different letters on the columns indicate significant differences (*P* < 0.05). A significant difference between values was determined by the one-way ANOVA with the Duncan test.

**Figure 3:** Plasma concentration of triglyceride and cholesterol in the rats fed on experimental treatments. Different letters on the columns indicate significant differences (*P* < 0.05). Significant difference between values was determined by the one-way ANOVA with Duncan test.

**Figure 4:** Plasma alkaline phosphatase and amylase activities in the rats fed on experimental treatments. Different letters on the columns indicate significant differences (*P* < 0.05). Significant difference between values was determined by one-way ANOVA with Duncan test.

**Figure 5:** Effects of oral administration of GP peptides on plasma ALT, AST, and AST/ALT ratio in the rats fed on experimental treatments. Different letters on the columns indicate significant differences (*P* < 0.05). Significant differences between values were determined by one-way ANOVA with the Duncan test.

**Figure 6:** Effects of oral administration of GP peptides on plasma concentration of proinflammatory cytokines (TNF-*α*, IL-6) in the rats fed on experimental treatments. Different letters on the columns indicate significant differences (*P* < 0.05). Significant differences between values were determined by one-way ANOVA with the Duncan test.

**Figure 7:** Fasting glucose, insulin, glucose tolerance, and HOMA-IR values in the rats fed on HFD and GP peptides after 70 days of the experiment period. Different letters on the columns indicate significant differences (*P* < 0.05). Significant differences between values were determined by one-way ANOVA with the Duncan test.

**Figure 8:** Expression of autophagy genes (Becline 1, Atg7, LC3-ɪ, and P62) in the liver of the induced NAFLD rats. Different letters on the columns indicate significant differences (*P* < 0.05). Significant difference between values was determined by one-way ANOVA with the Duncan test.

**Figure 9:** Hematoxylin and eosin (H&E) staining of liver tissue sections from control (A1, A2), HFD (B1, B2), HFD + GP20 (C1, C2), and HFD + GP300 (D1, D2) (×400).

**Figure 10:** Sudan Black staining of liver tissue sections from control, HFD, HFD + GP20, and HFD + GP300 (left to right, respectively) (×400).

**Table 1:** Nucleotide sequence of primers used for PCR.

Gene	Primer	AT	bp
P62	F: GCTGCTCTCTTCAGGCTTACAG	53°C	22
	R: CCTGCTTCACAGTAGACGAAAG		

Beclin-1	F: AGCACGCCATGTATAGCAAAGA	51°C	22
	R: GGAAGAGGGAAAGGACAGCAT		

Atg7	F: AGCCTGTTCATCCAAAGTTCT	46°C	21
	R: CTGTGGTTGCTCAGACGGT		

LC3-I	F: GATGTCCGACTTATTCGAGAGC	46°C	22
	R: TTGAGCTGTAAGCGCCTTCTA		

GAPDH	F: AAGGTCATCCATGACAACTT	58°C	20
	R: GGCCATCCACAGTCTTCTGG		

**Table 2:** The effects of GP peptides on weight gain and relative weight of the liver in NAFLD-induced rats after 70 days of the experiment period.

	Control	HFD	HFD + GP20	HFD + GP300
Weight gain (g)	62.6 ± 11.2	53.6 ± 10.4	59.3 ± 11.5	63.0 ± 10.6
Liver weight (g)	2.8 ± 0.2	3.2 ± 0.2	2.6 ± 0.2	3.1 ± 0.6

Data are expressed as mean ± SD (*n* = 6 per treatment).Different letters within a row indicate significant differences (*P* < 0.05).

## Data Availability

The data are available upon request to the corresponding author.

## References

[1] Carabelli J., Burgueno A. L., Rosselli M. S. (2011). High fat diet‐induced liver steatosis promotes an increase in liver mitochondrial biogenesis in response to hypoxia. *Journal of Cellular and Molecular Medicine*.

[2] Erdmann K., Grosser N., Schipporeit K., Schröder H. (2006). The ACE inhibitory dipeptide Met-Tyr diminishes free radical formation in human endothelial cells via induction of heme oxygenase-1 and ferritin. *Journal of Nutrition*.

[3] Gao J., Song J., Du M., Mao X. (2019). Bovine *α*-lactalbumin hydrolysates (*α*-LAH) attenuate high-fat diet induced nonalcoholic fatty liver disease by modulating hepatic lipid metabolism in C57BL/6J mice. *Journal of Functional Foods*.

[4] Venugopal V. (2008). *Marine Products for Healthcare: Functional and Bioactive Nutraceutical Compounds from the Ocean*.

[5] Giri A., Ohshima T. (2012). Bioactive marine peptides: nutraceutical value and novel approaches. *Advances in Food & Nutrition Research*.

[6] Agyei D., Danquah M. K. (2012). Rethinking food-derived bioactive peptides for antimicrobial and immunomodulatory activities. *Trends in Food Science & Technology*.

[7] Tang W., Zhang H., Wang L., Qian H., Qi X. (2015). Targeted separation of antibacterial peptide from protein hydrolysate of anchovy cooking wastewater by equilibrium dialysis. *Food Chemistry*.

[8] Athmani N., Dehiba F., Allaoui A. (2015). Sardina pilchardus and Sardinella aurita protein hydrolysates reduce cholesterolemia and oxidative stress in rat fed high cholesterol diet. *Journal of Experimental and Integrative Medicine*.

[9] Erdmann K., Cheung B. W., Schröder H. (2008). The possible roles of food-derived bioactive peptides in reducing the risk of cardiovascular disease. *The Journal of Nutritional Biochemistry*.

[10] Vik R., Tillander V., Skorve J. (2015). Three differently generated salmon protein hydrolysates reveal opposite effects on hepatic lipid metabolism in mice fed a high-fat diet. *Food chemistry*.

[11] Huang F., Wang J., Yu F. (2018). Protective effect of meretrix meretrix oligopeptides on high-fat-diet-induced non-alcoholic fatty liver disease in mice. *Marine Drugs*.

[12] Abbate J. M., Macrì F., Capparucci F. (2020). Administration of Protein Hydrolysates from Anchovy (Engraulis Encrasicolus) waste for twelve weeks decreases metabolic dysfunction-associated fatty liver disease severity in ApoE–/–Mice. *Animals*.

[13] FAO (2018). *Global Aquaculture Production*.

[14] Sachindra N., Bhaskar N., Mahendrakar N. (2006). Recovery of carotenoids from shrimp waste in organic solvents. *Waste Management*.

[15] Nikoo M., Xu X., Regenstein J. M., Noori F. (2020). Autolysis of Pacific white shrimp (Litopenaeus vannamei) processing by-products: Enzymatic activities, lipid and protein oxidation. *Food Bioscience*.

[16] Nasri R., Abdelhedi O., Jemil I. (2015). Ameliorating effects of goby fish protein hydrolysates on high-fat-high-fructose diet-induced hyperglycemia, oxidative stress and deterioration of kidney function in rats. *Chemico-Biological Interactions*.

[17] Zhao Y.-R., Wang D., Liu Y., Shan L., Zhou J.-L. (2016). The PI3K/Akt, p38MAPK, and JAK2/STAT3 signaling pathways mediate the protection of SO2 against acute lung injury induced by limb ischemia/reperfusion in rats. *The Journal of Physiological Sciences*.

[18] Sun Y., Oberley L. W., Li Y. (1988). A simple method for clinical assay of superoxide dismutase. *Clinical Chemistry*.

[19] Lowry O., Rosebrough N., Farr A. L., Randall R. (1951). The Lowry protein assay. *Journal of Biological Chemistry*.

[20] Boonloh K., Kukongviriyapan V., Kongyingyoes B., Kukongviriyapan U., Thawornchinsombut S., Pannangpetch P. (2015). Rice bran protein hydrolysates improve insulin resistance and decrease pro-inflammatory cytokine gene expression in rats fed a high carbohydrate-high fat diet. *Nutrients*.

[21] Matthews D. R., Hosker J. P., Rudenski A. S., Naylor B. A., Treacher D. F., Turner R. C. (1985). Homeostasis model assessment: insulin resistance and *β*-cell function from fasting plasma glucose and insulin concentrations in man. *Diabetologia*.

[22] Akbar Gharehbagh S., Tolouei Azar J., Razi M. (2021). ROS and metabolomics-mediated autophagy in rat’s testicular tissue alter after exercise training; Evidence for exercise intensity and outcomes. *Life Sciences*.

[23] Brunt E. M., Janney C. G., Di Bisceglie A. M., Neuschwander-Tetri B. A., Bacon B. R. (1999). Nonalcoholic steatohepatitis: a proposal for grading and staging the histological lesions. *American Journal of Gastroenterology*.

[24] Amini Sarteshnizi R., Sahari M. A., Ahmadi Gavlighi H., Regenstein J. M., Nikoo M., Udenigwe C. C. (2021). Influence of fish protein hydrolysate-pistachio green hull extract interactions on antioxidant activity and inhibition of *α*-glucosidase, *α*-amylase, and DPP-IV enzymes. *LWT*.

[25] Das J., Ghosh S., Sil P. C. (2020). Taurine and cardiac oxidative stress in diabetes. *Diabetes*.

[26] Sampath W. W. H. A., Rathnayake R. M. D. S., Yang M., Zhang W., Mai K. (2020). Roles of dietary taurine in fish nutrition. *Marine Life Science & Technology*.

[27] Drotningsvik A., Mjøs S. A., Høgøy I., Remman T., Gudbrandsen O. A. (2015). A low dietary intake of cod protein is sufficient to increase growth, improve serum and tissue fatty acid compositions, and lower serum postprandial glucose and fasting non-esterified fatty acid concentrations in obese Zucker fa/fa rats. *European journal of nutrition*.

[28] Drotningsvik A., Mjos S. A., Pampanin D. M. (2016). Dietary fish protein hydrolysates containing bioactive motifs affect serum and adipose tissue fatty acid compositions, serum lipids, postprandial glucose regulation and growth in obese Zucker fa/fa rats. *British Journal of Nutrition*.

[29] Konrad D., Rudich A., Schoenle E. J. (2007). Improved glucose tolerance in mice receiving intraperitoneal transplantation of normal fat tissue. *Diabetologia*.

[30] Mlinar B., Marc J., Janež A., Pfeifer M. (2007). Molecular mechanisms of insulin resistance and associated diseases. *Clinica Chimica Acta*.

[31] Noguchi N., Yanagita T., Rahman S. M., Ando Y. (2016). Chlorella protein hydrolysate attenuates glucose metabolic disorder and fatty liver in high-fat diet-induced obese mice. *Journal of Oleo Science*.

[32] Yki-Järvinen H. (2014). Non-alcoholic fatty liver disease as a cause and a consequence of metabolic syndrome. *Lancet Diabetes & Endocrinology*.

[33] Aloysius T. A., Carvajal A., Slizyte R., Skorve J., Berge R., Bjorndal B. (2018). Chicken protein hydrolysates have anti-inflammatory effects on high-fat diet induced obesity in mice. *Medicine (Baltimore)*.

[34] Chiang W.-D., Huang C. Y., Paul C. R., Lee Z.-Y., Lin W.-T. (2016). Lipolysis stimulating peptides of potato protein hydrolysate effectively suppresses high-fat-diet-induced hepatocyte apoptosis and fibrosis in aging rats. *Food & Nutrition Research*.

[35] Lemus-Conejo A., Grao-Cruces E., Toscano R. (2020). A lupine (Lupinus angustifolious L.) peptide prevents non-alcoholic fatty liver disease in high-fat-diet-induced obese mice. *Food & Function*.

[36] Lavallard V. J., Gual P. (2014). Autophagy and non-alcoholic fatty liver disease. *BioMed Research International*.

[37] Alam M., Kauter K., Brown L. (2013). Naringin improves diet-induced cardiovascular dysfunction and obesity in high carbohydrate, high fat diet-fed rats. *Nutrients*.

[38] Grundy S. M. (2004). Obesity, metabolic syndrome, and cardiovascular disease. *Journal of Clinical Endocrinology & Metabolism*.

[39] da Cunha N. V., Pinge-Filho P., Panis C. (2014). Decreased endothelial nitric oxide, systemic oxidative stress, and increased sympathetic modulation contribute to hypertension in obese rats. *American Journal of Physiology - Heart and Circulatory Physiology*.

[40] Chitapanarux T., Tienboon P., Pojchamarnwiputh S., Leelarungrayub D. (2009). Open‐labeled pilot study of cysteine‐rich whey protein isolate supplementation for nonalcoholic steatohepatitis patients. *Journal of Gastroenterology and Hepatology*.

[41] Marnett L. J. (1999). Lipid peroxidation—DNA damage by malondialdehyde. *Mutation Research, Fundamental and Molecular Mechanisms of Mutagenesis*.

[42] Mamun M. A. A., Faruk M., Rahman M. M. (2019). High carbohydrate high fat diet induced hepatic steatosis and dyslipidemia were ameliorated by Psidium guajava leaf powder supplementation in rats. *Evidence-based Complementary and Alternative Medicine*.

[43] Rahman M. M., Alam M. N., Ulla A. (2017). Cardamom powder supplementation prevents obesity, improves glucose intolerance, inflammation and oxidative stress in liver of high carbohydrate high fat diet induced obese rats. *Lipids in Health and Disease*.

[44] Umayaparvathi S., Meenakshi S., Vimalraj V., Arumugam M., Sivagami G., Balasubramanian T. (2014). Antioxidant activity and anticancer effect of bioactive peptide from enzymatic hydrolysate of oyster (Saccostrea cucullata). *Biomedicine & Preventive Nutrition*.

[45] Sarmadi B. H., Ismail A. (2010). Antioxidative peptides from food proteins: a review. *Peptides*.

[46] Taliercio J. J., Schold J. D., Simon J. F. (2013). Prognostic importance of serum alkaline phosphatase in CKD stages 3-4 in a clinical population. *American Journal of Kidney Diseases*.

[47] Shariatifar B., Khodadoostan M., Motamedi N., Abdolahi H. (2016). Comparison of liver enzymes level and sonographic findings value with liver biopsy findings in nonalcoholic fatty liver disease patients. *Advanced Biomedical Research*.

[48] Mao Y. Q., Yu F., Wang J., Guo C., Fan X. (2016). Autophagy: a new target for nonalcoholic fatty liver disease therapy. *Hepatic Medicine: Evidence and Research*.

[49] Huang F., Wang J., Yu F. (2018). Protective Effect of Meretrix meretrix Oligopeptides on high-fat-diet-induced non-alcoholic fatty liver disease in mice. *Mar Drugs*.

[50] Singh R., Kaushik S., Wang Y. (2009). Autophagy regulates lipid metabolism. *Nature*.

[51] Ryter S. W., Mizumura K., Choi A. M. K. (2014). The impact of autophagy on cell death modalities. *International Journal of Cell Biology*.

[52] Runwal G., Stamatakou E., Siddiqi F. H., Puri C., Zhu Y., Rubinsztein D. C. (2019). LC3-positive structures are prominent in autophagy-deficient cells. *Scientific Reports*.

[53] Liu W. J., Ye L., Huang W. F. (2016). p62 links the autophagy pathway and the ubiqutin–proteasome system upon ubiquitinated protein degradation. *Cellular and Molecular Biology Letters*.

[54] Jain A., Lamark T., Sjottem E. (2010). p62/SQSTM1 is a target gene for transcription factor NRF2 and creates a positive feedback loop by inducing antioxidant response element-driven gene transcription. *Journal of Biological Chemistry*.

[55] Scherz‐Shouval R., Shvets E., Fass E., Shorer H., Gil L., Elazar Z. (2007). Reactive oxygen species are essential for autophagy and specifically regulate the activity of Atg4. *The EMBO Journal*.

